# Micro Expression Recognition via Dual-Stream Spatiotemporal Attention Network

**DOI:** 10.1155/2021/7799100

**Published:** 2021-08-17

**Authors:** Yan Wang, Yikun Huang, Can Liu, Xiaoying Gu, Dandan Yang, Shuopeng Wang, Bo Zhang

**Affiliations:** ^1^College of Information Engineering, Tianjin University of Commerce, Tianjin 300134, China; ^2^Concord University College of Fujian Normal University, Fuzhou, Fujian 350117, China; ^3^School of Artificial Intelligence, Hebei University of Technology, Tianjin 300401, China

## Abstract

Microexpression can manifest the real mood of humans, which has been widely concerned in clinical diagnosis and depression analysis. To solve the problem of missing discriminative spatiotemporal features in a small data set caused by the short duration and subtle movement changes of microexpression, we present a dual-stream spatiotemporal attention network (DSTAN) that integrates dual-stream spatiotemporal network and attention mechanism to capture the deformation features and spatiotemporal features of microexpression in the case of small samples. The Spatiotemporal networks in DSTAN are based on two lightweight networks, namely, the spatiotemporal appearance network (STAN) learning the appearance features from the microexpression sequences and the spatiotemporal motion network (STMN) learning the motion features from optical flow sequences. To focus on the discriminative motion areas of microexpression, we construct a novel attention mechanism for the spatial model of STAN and STMN, including a multiscale kernel spatial attention mechanism and global dual-pool channel attention mechanism. To obtain the importance of each frame in the microexpression sequence, we design a temporal attention mechanism for the temporal model of STAN and STMN to form spatiotemporal appearance network-attention (STAN-A) and spatiotemporal motion network-attention (STMN-A), which can adaptively perform dynamic feature refinement. Finally, the feature concatenate-SVM method is used to integrate STAN-A and STMN-A to a novel network, DSTAN. The extensive experiments on three small spontaneous microexpression data sets of SMIC, CASME, and CASME II demonstrate the proposed DSTAN can effectively cope with the recognition of microexpressions.

## 1. Introduction

Microexpression is a kind of spontaneous facial expression that can reveal the real emotion that people try to hide. The duration of microexpression is short, only lasting 1/25 s∼1/5 s [1]. And the muscle movement caused by microexpression only appears in a small area of the face, which limits the performance of recognizing microexpression to a certain extent. In recent years, a large number of automatic recognition methods have emerged, which greatly improve the application feasibility of microexpression. At present, microexpression recognition has a wide application prospect in the police interrogation, clinical diagnosis, depression analysis, and other fields [2–5].

In the microexpression recognition procedures, feature extraction is the critical step and researchers strive to seek the reprehensive methods. LBP-TOP (local binary pattern with three orthogonal planes) [6] is a typical texture feature-based method for microexpression recognition and taken as the baseline of handcraft methods. Due to its shortcomings of sensitivity and sparse sampling, there are many improved methods, such as LBP-SIP (local binary pattern with six intersection points) [7], STLBP-IP (spatial-temporal local binary pattern with integral projection) [8], STCLQP (spatial-temporal completed local quantized patterns) [9], and LCBP (local cube binary pattern) [10], to enhance the robustness of the features.

Furthermore, the optical flow-based methods exploit the changes of the pixels in the time domain and the correlations between the sequence frames to mine the correspondence in adjacent frames. The classical approaches include MDMO (main directional mean optical flow feature) [11], which can identify microexpression by locating the main direction of the face block and calculating the average optical flow of the face block. MDMO is characterized by simple calculation and small feature dimensions, but it is easy to miss the low-level manifold structure. Based on MDMO, researchers have proposed various improved methods, such as FDM (Facial Dynamics Map) [12], Sparse MDMO [13], and Bi-WOOF (Bi-Weighted Oriented Optical Flow) [14], to extract the motion features of microexpression more effectively.

Although the texture-based and motion-based methods solved the recognition problems to a certain extent, the features got by these handcraft methods need artificial design and it is difficult to automatically extract discriminative information using these methods. Latterly, deep learning approaches, such as CNNs (convolutional neural networks) and LSTM (long short-term memory), have shown their powerful abilities in many fields. These methods avoid the tedious handcraft feature design and can automatically capture the subtle changes of microexpressions. Kim et al. [15] adopted the two-step model CNN-LSTM to recognize microexpressions. They utilize CNNs to extract the spatial features of a frame and then put the features into LSTM to learn the temporal information of the microexpression sequence. Li et al. [16] proposed 3D-FCNN to extract the deep spatiotemporal features to identify the microexpression. Khor et al. [17] presented the method of ELRCN-TE.

They fused the original sequence, optical flow sequence, and optical strain sequence of microexpression and adopted VGG-LSTM to extract the spatiotemporal features of microexpression. Xia et al. [18] designed STRCN by fusing the appearance and geometry features to extend the connectivity of convolutional networks in the time domain. However, these methods do not consider the complementarity of high-level, low-level networks and the contribution of various image pixels to recognize microexpressions.

Since the attention mechanism has been successfully applied to many tasks, Chu et al. [19] combined CNN and multicontext attention to form an end-to-end framework for human pose estimation. Zhang et al. [20] used progressive attention to guide RNN for detecting salient objects. Due to the subtlety and short duration of microexpression, Yang et al. [21] proposed MERTA by utilizing three attention mechanisms to construct feature maps. Nevertheless, these attention-based methods mostly handle multilevel features without distinction, ignoring the differences between high-level and low-level network features and the intensity difference between the microexpression frames.

Inspired by these works, this paper constructs a dual-stream spatiotemporal network, DSTAN, by using STAN-A (STAN with attention mechanism) to extract appearance features and STMN-A (STMN with attention mechanism) to get motion features of microexpression sequences, respectively. Considering the small size of the microexpression data set and the low motion intensity of microexpression, this paper designs two lightweight networks, STAN and STMN, to extract subtle microexpression features. Besides, to focus on the key regions of microexpression, we introduce two attention mechanisms to the spatial model of STAN and STMN: the multiscale kernel spatial attention mechanism is applied to get the detailed low-level features, and the global dual-pool channel attention mechanism is applied to obtain the high-level features. Given the importance of different frames, the temporal attention mechanism is employed in the temporal model of STAN and STMN, so that the model can learn more representative features. Finally, the feature concatenate-SVM method is used to integrate the dual-stream networks STAN-A and STMN-A, which integrate the two spatiotemporal networks STAN and STMN and attention mechanisms to realize the task of microexpression recognition.

## 2. Proposed Method

The overall framework of DSTAN is shown in Figure 1. STAN-A extracts spatiotemporal appearance features from the original microexpression sequence, and STMN-A extracts the spatiotemporal motion features from the optical flow sequence to describe the subtle motion changes of the microexpression. STAN and STMN are two networks that extract appearance features and motion features of microexpression, respectively. The multiscale kernel spatial attention and global dual-pool channel attention are introduced into the spatial model of STAN and STMN to extract the refined spatial features of the microexpression. Then, the spatial features are input into the temporal model of STAN and STMN to get the spatiotemporal features of the microexpression. Finally, the STAN with attention (STAN-A) and the STMN with attention (STMN-A) are integrated by feature concatenate-SVM to obtain the predicted category of the microexpression.

### 2.1. Image Preprocessing

First, we carry on face detection for each frame and locate the feature points. Based on these key points, the face region is blocked. To remove the impacts of head movements on recognition, we conduct facial alignment on the images to eliminate the differences of faces and sequences in the expressionless state. Furthermore, the aligned frames are normalized in the spatial domain, that is, to maintain the size of the frame uniformity. Generally, the length of the microexpression sequence is different, but the deep learning network usually needs a fixed length of the input dimension in the training stage. Therefore, it is necessary to normalize the microexpression sequence in the time domain. We use the TIM (temporal interpolation model) [22] to handle the original sequence to a fixed number of frames, and the sequence with a fixed length is taken as the input of STAN-A. The optical flow information between two adjacent frames is calculated from the original sequence, and the obtained fixed-length optical flow sequence is set as the input of STMN-A.

### 2.2. STMN

The spatial model of STMN is designed as a shallow network. Firstly, we use a kernel of 3×3 to conduct the convolution operations on the input optical flow sequence to extract local features. To avoid losing the edge information, zero padding is performed before convolution operation, and batch normalization [23] is used after convolution to accelerate the training speed of the model. We utilize ReLU as an activation function to enhance the nonlinear expression ability of the network. Each convolution layer is connected with a maximum pooling layer, and downsampling is performed under the condition of a 2 × 2 neighborhood and 2-step size. The local microexpression features are obtained after five times of convolution and pooling operation. Then, we adopt the GAP (global average pooling) to integrate these features and obtain the spatial features.

The temporal model of STMN is to obtain dynamic information between frames. The spatial feature vector describing the motion information of the microexpression obtained by the spatial model is input into the single-layer LSTM to learn the correlation between frames and obtain the feature vector *v*_*i*_ of each microexpression sequence. Then, the feature vectors are aggregated through a temporal average pooling operation to obtain the spatiotemporal feature *f* of the whole sequence:

(1) $$\begin{array}{c} f=\frac{1}{t}\sum_{i=1}^{t}v_{i}, \end{array}$$

where *i* = 1,2,…, *t*, and *t* represents the number of frames. Finally, the fully connected layer is applied to map the feature space to the label space through linear transformation, and softmax is used to map the output to (0, 1) to obtain the category of microexpression.

### 2.3. STAN

Considering that the features in different levels are complementary, we design the spatial model for STAN fusing high-level and low-level features, and the model can learn both deep semantic and low texture features, as the LHFN (low high feature fusion network) module in Figure 1 shows. In CNNs, different convolution layers learn different features; the third convolution layers can learn the low-level texture features [24], which play an important role in recognizing microexpression, so we fuse it with the last layer, which can learn the high-level semantic features to realize the high-level and low-level networks. The implementation of LHFN is based on the convolution calculation with a convolution kernel of 1 × 1 on the high-level feature map and low-level feature map to introduce more nonlinear relations. Then, we apply the GAP layer to obtain global low-level texture features and high-level semantic features. Finally, the high-level and low-level features are fused by a feature concatenate mode to obtain the spatial features describing the appearance information of each frame. The temporal model of STAN is the same as the temporal structure of STMN.

### 2.4. Attention Mechanism for Spatial Model

The existing microexpression recognition approaches handle the contribution of each pixel in the image or frame equally. However, the microexpression mainly appears in specific parts of the face, such as eyes, eyebrows, and mouth. According to the feature differences of the low-level and high-level networks, we introduce a novel attention mechanism to the spatial domain model, which is composed of a multiscale kernel spatial attention mechanism and a global dual-pool channel attention mechanism.

We introduce the multiscale kernel spatial attention to the low-level network and the global dual-pool channel attention to the high-level network to make the network focus on these significant motion areas.

#### 2.4.1. Multiscale Kernel Spatial Attention Mechanism

The low-level network extracts the texture, edge, contour, and other low-level visual features of microexpression, and this information has almost no difference in different channels. Therefore, we apply the multiscale kernel spatial attention to the low-level network to effectively distinguish each pixel in the spatial domain. The implementation process is shown in Figure 2, and the calculating processes are as follows:

Given the low-level feature map *F*^*l*^ ∈ ℝ^*C*×*H*×*W*^, *C* is the number of feature channels, and *H* and *W* are the height and width of the feature map, respectively. The first step is to conduct convolution operations Conv_*m*_^*n*×*n*^() on feature map *F*^*l*^ by the convolution kernel *n* of 1 × 1, 3 × 3, and 5 × 5 to extract multiscale feature, and the spatial feature matrix of different scales *S*_1_ ∈ ℝ^1×*H*×*W*^, *S*_2_ ∈ ℝ^1×*H*×*W*^, and *S*_3_ ∈ ℝ^1×*H*×*W*^ are obtained:

(2) $$\begin{array}{c} S_{1}={\text{Conv}}_{1}^{1\times 1}\left(F^{l}\right),\\ S_{2}={\text{Conv}}_{2}^{3\times 3}\left(F^{l}\right),\\ S_{3}={\text{Conv}}_{3}^{5\times 5}\left(F^{l}\right). \end{array}$$

Then, we fuse *S*_1_, *S*_2_, and *S*_3_ by concatenate mode and conduct convolution operation by the convolution kernel of 1 × 1 to obtain spatial features. Afterward, we obtain the weight *SA* ∈ ℝ^1×*H*×*W*^ of spatial attention by normalizing as below:

(3) $$\begin{array}{c} SA=\sigma \left({\text{Conv}}_{4}^{1\times 1}\left(S_{1},S_{2},S_{3}\right)\right). \end{array}$$

Finally, we multiply *SA* with *F*^*l*^ and get the refined spatial attention feature map *F*_*S*_ ∈ ℝ^*C*×*H*×*W*^:

(4) $$\begin{array}{c} F_{S}=SA⊗F^{l}, \end{array}$$

where ⊗ denotes the matrix multiplied by elements, and *σ* is the sigmoid function.

#### 2.4.2. Global Dual-Pooling Channel Attention Mechanism

A high-level network extracts high-level semantic feature information, and different feature channels have different responses to different semantic features [25]. Max-pooling can preserve more texture information, average pooling can retain more local information, and utilizing maximum pooling and average pooling at the same time can greatly improve the network's presentation capabilities [26]. Consequently, we present the global dual-pooling channel attention mechanism to the high-level network, which combines the max-pooling operation with average pooling operation effectively. This kind of attention mechanism automatically obtains the contribution of each feature channel. Through this attention mechanism, the effective features are enhanced while the features of little matter are suppressed. The global dual-pooling channel attention mechanism is shown in Figure 3.

The calculation process is as follows: given the input high-level feature graph *F*^*h*^ ∈ ℝ^*C*×*H*×*W*^, *C* is the number of feature channels, and *H* and *W* are the height and width of the feature map, respectively. Firstly, we conduct GAP and GMP (global max-pooling) operation on *F*^*h*^ to aggregate the spatial information of the feature map and obtain the global average pooling feature vector *F*_*C*_^*GMP*^ ∈ ℝ^*C*×1×1^ and global max-pooling feature vector *F*_*C*_^*GAP*^ ∈ ℝ^*C*×1×1^. Then, we use two consecutive full-connection layers *FC*_1_ and *FC*_2_ to fine-tune the parameters adaptively to learn the dependence and correlation of different channels. To reduce the model complexity, we set the number of units in *FC*_1_ as *C*/*r*, where *r* is the compression ratio, and the number of units in *FC*_2_ as *C*. Through a full-connection layer, we can get two-channel feature vectors *C*_1_∈ℝ^*C*×1×1^ and *C*_2_∈ℝ^*C*×1×1^:

(5) $$\begin{array}{c} C_{1}=FC_{2}\left(\delta \left(FC_{1}\left(GAP\left(F^{h}\right)\right)\right)\right)=w_{2}\left(\delta \left(w_{1}\left(F_{C}^{GAP}\right)+b_{1}\right)\right)+b_{2},\\ C_{2}=FC_{2}\left(\delta \left(FC_{1}\left(GMP\left(F^{h}\right)\right)\right)\right)=w_{2}\left(\delta \left(w_{1}\left(F_{C}^{GMP}\right)+b_{1}\right)\right)+b_{2}. \end{array}$$

Next, we merge *C*_1_ and *C*_2_ through element summation. The weight *CA*∈ℝ^*C*×1×1^ of channel attention can be got by normalizing as below:

(6) $$\begin{array}{c} CA=\sigma \left(C_{1}⊕C_{2}\right). \end{array}$$

Finally, we obtain the refined feature map *F*_*C*_ ∈ ℝ^*C*×*H*×*W*^ of channel attention by multiplying *CA* and *F*^*h*^:

(7) $$\begin{array}{c} F_{C}=CA⊗F^{h}, \end{array}$$

where *δ* denotes the ReLU activation function, *σ* denotes the sigmoid function, ⊗ indicates that vectors are added, *w*_1_ and *w*_2_ are the weight of *FC*_1_ and *FC*_2_, and *b*_1_ and *b*_2_ are the offsets, respectively.

### 2.5. Attention Mechanism for Temporal Model

This paper introduces another attention mechanism into the temporal model so that the model can learn automatically and distinguish the important frames in the microexpression sequence. The attention mechanism for the temporal model is shown in Figure 4. The feature vector of each frame obtained by the spatial model is input into the model, and an attention weight representing the importance of the frame is calculated. Specifically, for the spatial feature vector *S*_*i*_′ corresponding to the *i*-*th* frame, we use the sigmoid function to obtain the attention weight *r*_*i*_ for each frame and then perform a weighted operation on the obtained attention weight to get the feature vector *S*_*i*_′ of each frame.

(8) $$\begin{array}{c} S_{i}^{\prime }=S_{i}r_{i}, \end{array}$$

where *i* = 1, 2,…, *t*, and *t* represents the number of frames. The weighted spatial feature vector of each frame *S*_*i*_′ is input into the temporal models of STAN and STMN, respectively, to obtain the refined spatiotemporal appearance features and spatiotemporal motion features of a sequence.

### 2.6. Model Integration

We integrate STAN-A and STMN-A by the feature concatenate-SVM method. Firstly, the SVC (support vector classification) is initialized with a linear kernel function to define the classifier. Then, the linear multivariate classifier is trained by the microexpression data in the training set, as shown in Equation (9):

(9) $$\begin{array}{c} \left\|X:f\left(p_{i},q_{i}\right),Y\right\|⟶SVM, \end{array}$$

where *p*_*i*_ and *q*_*i*_ are the outputs of STAN-A and STMN-A, respectively, and *f* (*p*_*i*_, *q*_*i*_) is the cascaded results, *X* denotes the features of the classifier, and *Y* represents the feature label.

## 3. Results and Discussion

### 3.1. Data Sets

To evaluate the performance of the proposed framework, we conduct experiments on three spontaneous microexpression data sets: SMIC (Spontaneous Micro-Expression Database) [27] CASME(Chinese Academy of Sciences Micro-Expression) [28], and CASME II [29]. SMIC contains three categories of microexpressions: positive (51), negative (70), and surprise (43), and a total of 164 samples from 16 subjects. In CASME, 172 samples of 19 subjects' microexpression sequences are collected and divided into 4 categories, that is, tense (70), expression (38), distinct (44), and surprise (20). There are 246 samples of 26 subjects on CASME II. There are divided into 5 categories: happiness (32), surprise (25), expression (27), distinct (63), and others (99).

### 3.2. Parameter Setting and Evaluation Criterion

We use the TIM model to normalize the length of the sequence to 9 frames, and the size of each frame is set to 224 × 224. In the global dual-pooling channel attention, the compression ratio *r* is set as 16. We adopt the cross-entropy loss function and Adam optimizer to train the model and set the batch size as 32.

To get a stable and reliable model, we conduct experiments on three microexpression data sets to evaluate the performance of the algorithm by using the LOSOCV, that is, all samples of a subject are taken as testing sets, and the rest are used as training sets.

We utilize accuracy, *F1-score*, precision, and recall as the evaluation criterion to evaluate the proposed model. Accuracy is the ratio of the correct predicting sample number to the total sample number:

(10) $$\begin{array}{c} \text{Accuracy}=\frac{TP+TN}{TP+FP+TN+FN}. \end{array}$$

*F1-Score* is the harmonic average of accuracy. *F1-Score, Precision*, and *Recall* can be calculated as follows [30]:

(11) $$\begin{array}{c} F1-\text{Score}=2\times \frac{\text{Precision}\times \text{Recall}}{\text{Precision}+\text{Recall}},\\ \text{Precision}=\frac{TP}{TP+FP},\\ \text{Recall}=\frac{TP}{TP+FN}, \end{array}$$

where *TP* (true positive) indicates the number of samples that positive is predicted as positive; *FP* (false positive) indicates the number of samples that negative is predicted as positive; *TN* (true negative) is the number of samples that negative is predicted as negative; and *FN* (false negative) is the number of samples that positive is predicted as negative.

### 3.3. Experimental Analysis

In this section, ablation experiments and performance verification are performed on the proposed DSTAN framework, and comparative experiments are conducted with state-of-the-arts.

#### 3.3.1. Comparison of Single Network with Dual-Stream Network

To verify the effectiveness of the dual-stream network, we compare the single-stream networks STAN-A and STMN-A with the dual-stream network DSTAN.  Table 1 shows the comparison results on three data sets. It can be seen that the performance of the dual-stream network DSTAN is better than that of STAN-A and STMN-A on three data sets. Specifically, compared with STAN-A and STMN-A, the accuracy of DSTAN is increased by 9.15% and 12.2% and *F1-score* is increased by 10.64% and 12.84% on SMIC. On CASME, the accuracy of DSTAN is increased by 11.05% and 12.79% and *F1-score* is increased by 12.47% and 13.97%. On CASME II, the accuracy of DSTAN is increased by 15.04% and 11.38% and *F1-score* is increased by 16.91% and 12.18%. The results show that the dual-stream network DSTAN outperforms the single-stream network, which can verify that DSTAN can make the model learn more discriminative features and improve the overall recognition performance.

Furthermore, we compare the recognition performance of each emotion on three data sets, as shown in Figure 5. On SMIC, as shown in Figure 5(a), STAN-A gets a higher recognition rate for “positive” but a poor result for “surprise”.

However, STMN-A has a good performance for “surprise” and low accuracy for “positive”. On CASME, as shown in Figure 5(b), STAN-A has a good performance on “disgust”, but it behaves poorly on “repression” and “surprise”. STMN-A has a good performance on these two emotions, but the “disgust” recognition result is lower. On CASME II, as can be seen from Figure 5(c), STAN-A and STMN-A are also complementary. Especially, the performance of STMN-A is lower than that of STAN-A in recognizing “disgust”, but DSTAN gets an ideal recognition result. Overall, STAN-A and STMN-A promote and complement each other in the recognition of emotions and DSTAN can get the best performance.

#### 3.3.2. Performance Verification of Different Modules

The proposed DSTAN combines high-level and low-level feature fusion modules (LHFN), spatial attention modules, and temporal attention modules based on the dual-stream network. To verify the effectiveness of different modules, ablation experiments are performed on the CASME II data set.

The basic model only contains the network, that is, the DSTAN removes the LHFN module, two spatial attention modules, and the temporal attention module. We compare the basic model with the models that are added LHFN module (basic model + LHFN), spatial attention modules (basic model + LHFN + SA), and temporal attention module (basic model + LHFN + SA + TA).  Table 2 shows the comparison result. It can be seen that by adding three modules to the basic model, the recognition result has been further improved. By adding the LHFN module, accuracy is increased by 1.62% and *F1-score* is increased by 1.67%. By adding the spatial attention modules, accuracy is increased by 4.07% and *F1-score* is increased by 3.64%. After adding the temporal attention module, accuracy is increased by 4.06% and *F1-score* is increased by 3.81%. The basic model + LHFN + SA + TA model (DSTAN) obtains the best recognition result and robustness. Therefore, these modules can improve the performance of recognizing microexpressions, which verifies the effectiveness of the modules. The LHFN module enables the model to learn discriminative semantic information of the microexpression sequence. The spatial attention module and temporal attention module can make the model learn more detailed and effective features.

#### 3.3.3. DSTAN Performance Analysis

We evaluate the DSTAN by using each subject as a testing set on three data sets. The experimental results are shown in Figure 6. The abscissa is the coding number of the subject, and the ordinate is the recognition accuracy of the subject. On SMIC, as shown in Figure 6(a), the DSTAN has good recognition results for most subjects, but the accuracy of the 3*rd* and the 4*th* subject is poor due to the action units of “negative” are similar to “surprise”, which makes them easy to be confused. On CASME, as shown in Figure 6(b), the accuracy rates on all of the 9 subjects are 100%, but the recognition result of the 1*st* subject is lower, it is because that “repression” is easily confused with “disgust” and “surprise”. As shown in Figure 6(c) on CASME II, the accuracy rate of the 16*th* subject is lower because there is a small number of this subject, only 4 sequences.

We calculated the confusion matrix of DSTAN on SMIC, CASME, and CASME II, as shown in Figure 7. On SMIC, as shown in Figure 7(a), the DSTAN performs well on identifying negative, positive, and superior emotions because the distribution of samples on this data set is relatively uniform. On CASME, as shown in Figure 7(b), the DSTAN gets a higher result for “tense”, “repression”, and “disgust”, but it is not good at recognizing “surprise” due to its small range of muscle motion. On CASME II, as shown in Figure 7(c), the DSTAN performs poorly in emotions “surprise” and “repression”. It is because “surprise,” “repression”, and “others” are easy to be confused as a result of the number of “others” has the largest data and the data set is unbalanced. The experimental results show that for the microexpression recognition task, the total number of samples of each emotion, the difference number of emotions, and the motion amplitude of microexpression are the important factors.

#### 3.3.4. Integration Mode Validation

Since most of the approaches adopt the weighted sum model to integrate, we compare it with the feature concatenate-SVM method.

The DSTAN with weighted sum integration mode is labeled as DSTAN-Average, and the DSTAN integrated by feature concatenate-SVM is marked as DSTAN-SVM.  Table 3 shows the comparison results on three microexpression data sets. The evaluation index *Precision* represents the discrimination ability of the model for negative samples, and *Recall* represents the recognition ability of the model for positive samples. As can be seen from Table 3, the performance of DSTAN-SVM is better than that of DSTAN-Average to a certain extent. On SMIC, CASME, and CASME II, the *Precision* of DSTAN-SVM is 3.29%, 2.94%, and 2.69% higher than that of DSTAN-Average, and *Recall* is increased by 4.46%, 2.39%, and 6.21%, respectively, which indicates that DSTAN-SVM has the discrimination ability for positive and negative samples. The accuracy of DSTAN-SVM is improved by 4.27%, 3.49%, and 4.47% compared with that of DSTAN-Average, and the *F1-score* is improved by 3.89%, 2.67%, and 4.68%, respectively, which indicates that DSTAN-SVM has better recognition performance and robustness.

#### 3.3.5. Comparison with State-of-the-Arts

The recognition performance of DSTAN is compared with some state-of-the-arts. The experimental results of the three data sets are shown in Table 4. LBP-TOP, LBP-SIP, STLBP-IP, STCLQP, and LCBP are texture feature-based methods. FDM, MDMO, Sparse MDMO, and Bi-WOOF are optical flow-based methods. 3D-FCNN, ELRCN-TE, STRCN, and MERTA are depth learning-based methods.

As can be seen from Table 4, on SMIC, the accuracy of DSTAN is 77.44%, which is 6.14% higher than the best method STRCN, and *F1-Score* is increased to 0.7783, which is 7.42% higher than Sparse MDMO. On CASME, the accuracy of DSTAN reaches 77.91%, which is 3.08% higher than Sparse MDMO, and *F1-Score* is 0.7516, which is 0.18% higher than Sparse MDMO. On CASME II, the Accuracy of DSTAN reaches 75.20%, which is 5.1% higher than the baseline method LCBP, and *F1-Score* is increased to 0.7283, which is 2.83% higher than LCBP. Experimental results show that the proposed DSTAN has better recognition performance than state-of-the-arts.

## 4. Conclusion

In this paper, we have presented a novel architecture for dynamic facial microexpression recognition combining deep and handcraft features, which can recognize the microexpressions with higher accuracy. Both the deep learning method and the handcraft method are fused to identify the microexpressions by learning features not only the tiny skin change but also the semantic properties from sequences. The approach successfully exploits spatial and temporal features of microexpression simultaneously. Particularly, the feature framework has been established to identify the dynamic microexpressions successfully by extracting robust features from data. In the end, we conduct extensive validation experiments to demonstrate the proposed method. The excessive experimental results showed that with an accuracy of 75.51% on SMIC, an accuracy of 81.26% on CASME_B, and an accuracy of 76.14% on CASME 2 in terms of the 5-class microexpression recognition, our framework can surpass other methods.

In the future, we aim to evaluate our approach on additional microexpression data sets. We also consider training our approach on cross-data-set experiments and explore the effective method to improve the recognition performance of microexpressions on action units.

## Figures and Tables

**Figure 1:** An illustration of the proposed DSTAN.

**Figure 2:** Multiscale kernel spatial attention mechanism.

**Figure 3:** Global dual-pool channel attention mechanism.

**Figure 4:** Attention mechanism for the temporal model.

**Figure 5:** Comparison of a single network with dual-stream network: (a) SMIE, (b) CASME, and (c) CASME II.

**Figure 6:** The performance of DSTAN for each subject: (a) SMIE, (b) CASME, and (c) CASME II.

**Figure 7:** Confusion matrix of DSTAN on three data sets: (a) SMIE, (b) CASME, and (c) CASME II.

**Table 1:** Comparison of single-stream with dual-stream network (F1 : *F1-score*).

Method	SMIC		CASME		CASME II	
	Accuracy	F1	Accuracy	F1	Accuracy	F1
STAN-A	0.683	0.672	0.669	0.627	0.602	0.559
STMN-A	0.652	0.649	0.651	0.612	0.638	0.607
DSTAN	0.774	0.778	0.779	0.752	0.752	0.728

**Table 2:** The influence of different modules on the network.

Method	CASME II	
	Accuracy	*F1*-*score*
Basic model	0.655	0.637
Basic model + LHFN	0.671	0.654
Basic model + LHFN + SA	0.711	0.690
Basic model + LHFN + SA + TA (DSTAN)	0.752	0.728

**Table 3:** Comparison results of two model integration methods.

Metrics	DSTAN-Average			DSTAN-SVM		
	SMIC	CASME	CASME II	SMIC	CASME	CASME II
Accuracy	0.73	0.74	0.71	0.77	0.78	0.75
Precision	0.75	0.73	0.74	0.79	0.76	0.77
Recall	0.73	0.72	0.63	0.77	0.75	0.70
*F1-score*	0.74	0.73	0.68	0.78	0.75	0.73

**Table 4:** Comparison of DSTAN with other approaches (F1 : *F1-Score*).

Method	SMIC		CASME		CASME II	
	Accuracy	F1	Accuracy	F1	Accuracy	F1
LBP-TOP [6]	0.44	0.41	0.37	0.33	0.47	0.35
LBP-SIP [7]	0.45	0.45	0.37	0.33	0.47	0.45
STLBP-IP [8]	0.58	—	—	—	0.56	—
STCLQP [9]	0.64	0.64	0.57	0.50	0.58	0.58
LCBP [10]	0.71	0.68	—	—	0.70	0.70
MDMO [11]	0.59	0.59	0.56	0.56	0.52	0.50
FDM [12]	0.55	0.54	0.56	0.49	0.46	0.41
Sparse MDMO [13]	0.71	0.70	0.75	0.75	0.67	0.69
Bi-WOOF [14]	0.62	0.62	—	—	0.59	0.61
CNN-LSTM [15]	—	—	—	—	0.61	—
3D-FCNN [16]	0.56	—	0.54	—	0.59	—
ELRCN-TE [17]	—	—	—	—	0.52	0.50
STRCN [18]	0.72	0.69	—	—	—	—
MERTA [21]	—	—	—	—	0.61	—
DSTAN	0.77	0.78	0.78	0.75	0.75	0.73

## Data Availability

All data included in this study are available upon request by contact with the corresponding author.

## References

[1] Yan W.-J., Wu Q., Liang J., Chen Y.-H., Fu X. (2013). How fast are the leaked facial expressions: the duration of micro-expressions. *Journal of Nonverbal Behavior*.

[2] Takalkar M. A., Xu M., Wu Q., Chaczko Z. (2018). A survey: facial micro-expression recognition. *Multimedia Tools and Applications*.

[3] Duan X., Dai Q., Wang X., Wang Y., Huo Z. (2016). Recognizing spontaneous micro-expression from eye region. *Neurocomputing*.

[4] Xue X., Chen J., Yao X. (2021). Efficient user involvement in semi-automatic ontology matching. *IEEE Transactions on Emerging Topics in Computational Intelligence*.

[5] Liu G., Chen X., Zhou R., Xu S., Chen Y.-C., Chen G. (2021). Social learning discrete particle swarm optimization based two-stage X-routing for IC design under intelligent edge computing architecture. *Applied Soft Computing*.

[6] Pfister T., Li X., Zhao G., Pietikäinen M. Recognizing spontaneous facial micro-expressions.

[7] Wang Y., See J., Phan R. C. W., Oh Y.-H. LBP with six intersection points: reducing redundant information in LBP-TOP for micro-expression recognition.

[8] Huang X., Wang S. J., Zhao G., Pietikäinen M. Facial micro-expression recognition using spatiotemporal local binary pattern with integral projection.

[9] Huang X., Zhao G., Hong X., Zheng W., Pietikäinen M. (2016). Spontaneous facial micro-expression analysis using Spatiotemporal completed local quantized patterns. *Neurocomputing*.

[10] Yu M., Guo Z. Q., Yu Y., Wang Y., Cen S. (2019). Spatiotemporal feature descriptor for micro-expression recognition using local cube binary pattern. *IEEE Access*.

[11] Liu Y., Zhang J., Yan W., Wang S., Zhao G., Fu X. (2016). A main directional mean optical flow feature for spontaneous micro-expression recognition. *IEEE Transactions on Affective Computing*.

[12] Xu F., Zhang J., Wang J. Z (2017). Micro expression identification and categorization using a facial dynamics map. *IEEE Transactions on Affective Computing*.

[13] Liu Y., Li B., Lai Y. (2018). Sparse MDMO: learning a discriminative feature for spontaneous micro-expression recognition. *IEEE Transactions on Affective Computing*.

[14] Liong S., See J., Wong K., Phan R. C. W. (2018). Less is more: micro-expression recognition from video using apex frame. *Signal Processing: Image Communication*.

[15] Kim D. H., Baddar W. J., Ro Y. M. Micro-expression recognition with expression-state constrained Spatial-temporal feature representations.

[16] Li J., Wang Y., See J. (2019). Micro-expression recognition based on 3d flow convolutional neural network. *Pattern Analysis & Applications*.

[17] Khor H. Q., See J., Phan R. C. W., Lin W. Enriched long-term recurrent convolutional network for facial micro-expression recognition.

[18] Xia Z., Hong X., Gao X., Feng X., Zhao G. (2020). Spatiotemporal recurrent convolutional networks for recognizing spontaneous micro-expressions. *IEEE Transactions on Multimedia*.

[19] Chu X., Yang W., Ouyang W., Ma C., Yuille A. L., Wang X. Multi-context attention for human pose estimation.

[20] Zhang X., Wang T., Qi J., Lu H., Wang G. Progressive attention guided recurrent network for salient object detection.

[21] Yang B., Cheng J., Yang Y., Zhang B., Li J. (2019). MERTA: micro-expression recognition with ternary attentions. *Multimedia Tools and Applications*.

[22] Zhou Z., Zhao G., Guo Y., Pietikainen M. (2012). An image-based visual speech animation system. *IEEE Transactions on Circuits and Systems for Video Technology*.

[23] Ioffe S., Szegedy C. Batch normalization: accelerating deep network training by reducing internal covariate shift.

[24] Zeiler M. D., Fergus R. Visualizing and understanding convolutional networks.

[25] Hu J., Shen L., Sun G., Wu E. Squeeze-and-Excitation networks.

[26] Woo S., Park J., Lee J., Kweon S. CBAM: convolutional block attention module.

[27] Li X, Pfister T, Huang X, Zhao J., Pietikainen M. A spontaneous micro-expression database: inducement, collection, and baseline.

[28] Yan W. J., Wu Q., Liu Y. J., Wang S. W., Fu X. CASME database: a dataset of spontaneous micro-expressions collected from neutralized faces.

[29] Yan W. J., Li X., Wang S. J. (2014). Casme II: an improved spontaneous micro-expression database and the baseline evaluation. *PLoS One*.

[30] Ngo A. C., Phan R. C., See J. Spontaneous subtle expression recognition: imbalanced databases and solutions.

